# Predictors and Preventive Strategies of Bleeding After Thyroid Surgery

This article has been retracted.

**DOI:** 10.7759/cureus.47575

**Published:** 2023-10-24

**Authors:** Mohsen Ezzy, Ehab Alameer

**Affiliations:** 1 Department of Surgery, College of Medicine, Jazan University, Jazan, SAU

**Keywords:** hemostasis, energy devices, hematoma, bleeding, thyroid surgery

## Abstract

Postoperative compressive neck hematoma occurs in approximately 0.1% to 1.7% of cases, most occurring within the first six hours after surgery. Thyroid pathology, patient predisposition, and surgical technique are major risk factors for postoperative hematoma. This narrative review describes current perspectives on predicting and preventing bleeding following thyroid surgery.

Predictors of bleeding after thyroid surgery include patient-related factors such as male sex and age, surgery-related factors like total thyroidectomy and operations for thyroid malignancy, and surgeon-related factors. Hemostasis is the primary focus after preserving critical structures in thyroid surgery.

The clamp-and-tie technique has been the standard method for dividing the thyroid gland's main vascular pedicles for many years. Bipolar electrocautery has been used for vessels of small size. However, advanced bipolar and ultrasound energy and hybrid devices are now available options that may reduce operative time without increasing costs or complications.

In cases where small bleeders close to critical structures are present and the clamp-and-tie technique is not feasible, hemostatic agents are commonly used. Drains do not appear to provide any significant benefits in preventing the sequelae of bleeding after thyroid surgery.

## Introduction and background

Post-thyroidectomy compressive neck hematoma is a significant concern for surgeons because it can cause severe and even life-threatening problems. Respiratory distress and airway compression can occur as a result of postoperative bleeding. Since the earliest attempts at performing this surgery, postoperative and intraoperative bleeding have historically been considered the most serious issues. In 1848, Dieffenbach described thyroid surgery as "one of the most perilous, thankless undertakings that, if not entirely forbidden, ought to be at least constrained." Shortly after, Gross (1866) wrote, "No sensible man will try to extirpate a goiter of the thyroid gland. Every move he makes will be surrounded by challenge, and a flood of blood will follow every stroke of his knife, and fortunate will he be if his victims live long." However, in the early 1900s, Emil Theodore Kocher was the one who first used precise surgical techniques and meticulous hemostasis to minimize the mortality rate to less than 0.5% in over 5,000 thyroidectomies [1].

The occurrence rate of postoperative compressive hematoma is approximately 0.1% to 1.7% [2]. In most cases, this happens within the first six hours after surgery and can be caused by numerous factors. Most studies report that approximately 20% of hematomas occur 6-24 hours after surgery, with almost no occurrences afterward [3]. Three categories of risk factors, namely surgical technique, patient predisposition, and thyroid pathology, are responsible for postoperative hematoma.

Recognizing factors that increase the risk of bleeding can help identify patients who require close monitoring and establish prevention methods. A Medline search revealed several articles on the incidence and risk factors of bleeding after thyroid surgery [4-8]. This review aims to outline strategies for predicting and preventing bleeding after thyroid surgery.

## Review

Pathophysiology of airway compromise and the importance of early recognition of post-thyroidectomy compressive hematoma

A postoperative hemorrhage in the neck can potentially contribute to airway compromise according to two potential mechanisms discussed in the literature: direct tracheal compression below the cricoid level or supraglottic edema secondary to venous compression.

An in vitro model [9] investigated whether the maximum possible pressure produced by a hematoma in the neck would be sufficient to directly compress the trachea, leading to tracheal compression. The study concluded that even pressure as high as 250 mmHg (systolic blood pressure) in neck hematomas would be insufficient to cause mechanical airway occlusion. A pilot study performed by Von Ahnen et al. [10] considered the use of continuous pressure measurement as a tool to detect postoperative bleeding after thyroid surgery. This study found that postoperative intra-cervical pressure ranged from sub-atmospheric to 7 mmHg at rest. In the case of rebleeding, the pressure rose to 36 mmHg.

Airway edema is described as the most likely mechanism for airway obstruction caused by a neck hematoma. According to Thakur et al., this mechanism entails impaired venous drainage from the head due to the hematoma's mass effect. The development of edema occurs within the arytenoid cartilages, the epiglottis, and the supraglottic structures [11,12].

Symptoms of bleeding are rarely investigated because they are affected by the amount of bleeding, the acquisition time, factors related to the patient, and the fact that these symptoms are not always found in all postoperative bleeding cases [6,13-18]. Discrete symptoms, such as cervical pressure and tightness, coughing, difficulty swallowing, change in voice, and restlessness, may be early symptoms of externally visible swelling of the neck preceded by a blood-soaked dressing or rapid filling or occlusion of wound drainage. Cervical swelling is not always a sign of significant bleeding and may also occur due to hemorrhage in the superficial subplatysmal layer. In contrast, even if there is no visible swelling in the neck, significant bleeding can be present in the deeper neck region, especially if the midline is completely closed [6,14-16]. Tachycardia, shortness of breath, hypotension, and stridor are symptoms and signs of significant bleeding that necessitate immediate reintervention. Hemoglobin levels and evaluation of coagulation parameters or bedside ultrasound examinations are not accurate diagnostic tools in postoperative cervical bleeding and should be omitted [19].

Risk factors and predictors of postoperative bleeding after thyroid surgery

Various researchers have discussed different risk factors for post-thyroidectomy bleeding. Thyroiditis, thyroid malignancy, and Graves' disease are frequently reported as important risk factors [13-18,20-25]. Table 1 summarizes possible risk factors for bleeding [19,26-27].

**Table 1:** Risk factors for bleeding after thyroid surgery

Category	Risk factor
Patient-related	Age
	Gender
	Haemophilia
	Von Willebrand’s disease
	Chronic renal failure
	Cirrhosis
	Anticoagulant medications
	Smoking
Thyroid pathology-related	Graves’ disease
	Toxic adenoma
	Toxic multinodular gland
	Intrathoracic goitres
	Recurrent goitres
	Malignancies
Surgical technique-related	Mode of access
	Strap muscle division
	Subplatysmal flaps
	Bilateral exploration
	Residual thyroid tissue
	Operation extent
	Previous thyroid surgery
	Neck dissection
Postoperative events-related	Cough
	Emesis
	Hypertension
Surgeon-related	The primary surgeon's experience
	Differences in the surgeon and hospital volumes

Patient-related, intervention-related, and surgeon-related factors may all play a role in predicting bleeding after thyroid surgery. Due to non-excludable interdependencies, a simple distinction between these risk factors is unlikely. Although the incidence of postoperative hemorrhage is relatively low in thyroid surgery, it may be associated with an increasing risk of hypoxic brain injury and asphyxia [27].

The published literature has evaluated the performance of individual surgeons as a relevant risk factor. It has been reported that surgeons significantly influence the incidence of postoperative bleeding, regardless of their training level. Lorenz et al. stated that there is a relationship between outcomes and surgeon volume in thyroid surgery. In addition to volume, cumulative experience is predicted to further improve the results [28].

According to Promberger et al., the quality of ligatures or clips used for hemostasis is important. Bleeding from blood vessels that were initially occluded but reopened by mechanical stress during extubation or due to postoperative vomiting and hypertension highlights the significant influence of anesthesiologists on the outcome. Performing the Valsalva maneuver before wound closure and maintaining acceptable mean blood pressure values aid in predicting and identifying bleeders [6].

Most studies in the literature have reported the use of antithrombotic medications to increase the incidence of rebleeding. Moreover, a history of bleeding associated with previous surgeries was found to be a significant risk factor [3,6,7,13,18,20,25,29-31]. Oltmann et al. reported in a recent retrospective review of a prospective endocrine surgery database that anticoagulants have a strong relationship with increased rates of hematoma formation in both thyroid and parathyroid surgery. Injectable anticoagulants specifically increase the risk of hematoma formation by 29 times. As a result, patients receiving anticoagulation therapy must be individually assessed for thromboembolic risk versus the risk of postoperative hematoma, and an effective perioperative anticoagulation strategy should be developed accordingly [32].

Preventive strategies

Preoperative Considerations

The perioperative management of anticoagulation involves balancing the risk of bleeding with the risk of thromboembolic events resulting from holding anticoagulants. It is also important to discuss the duration of the discontinuation of anticoagulation and the need for bridging therapy. In one study, out of 4663 participants who discontinued direct oral anticoagulants, one patient experienced a thrombotic cerebrovascular accident after thyroidectomy [33]. Although there is general guidance on quantifying bleeding risks and thromboembolism to guide perioperative preparation in general, this has not been explicitly addressed for neck endocrine surgery. Moreover, there is significant variation in practice among surgeons performing neck endocrine surgery [32].

We concur with Edafe et al. that further research is necessary to differentiate hematoma risks in patients undergoing neck endocrine surgery, with particular attention to anticoagulated patients, considering not only their risk of bleeding but also their thromboembolic events. Meanwhile, it is crucial to understand these risks in anticoagulated individuals so that the surgeon can adjust their surgical approach and have an open and honest preoperative discussion with the patient [33].

Intraoperative Considerations

Anesthesia: An important goal of anesthesia is to minimize postoperative nausea, as uncontrolled nausea can lead to retching and vomiting, which may cause bleeding in the surgical wound. Recent randomized trials have shown that the use of dexamethasone or pre-emptive antiemetic agents (such as droperidol) can alleviate postoperative nausea and vomiting [34,35]. Another crucial aspect of general anesthesia is ensuring a smooth emergence to reduce excessive coughing, which can increase the risk of postoperative bleeding. Various techniques have been suggested to minimize coughing during emergence, including deep extubation, the administration of dexmedetomidine, and the use of topical or intravenous lidocaine [2].

Surgical technique: For several years, the clamp-and-tie method has been the most common approach to controlling the main vascular pedicles of the thyroid gland. On the other hand, bipolar electrocautery has only been used for small vessels. Other hemostatic systems have been introduced and shown significant potential benefits in neck surgery, particularly thyroid surgery. These new instruments are often referred to as "energy devices" because they utilize various forms of energy. Examples of energy devices include advanced bipolar instruments (LigaSureTM Small Jaw Medtronic, a Covidien product, Minneapolis, MN, USA), ultrasound instruments (Harmonic Focus; Ethicon, Johnson & Johnson, Cincinnati, OH, USA), and hybrid devices (Thunderbeat by Olympus, Japan). Although these devices significantly increase tissue temperatures, the temperatures they reach are not as high as those achieved by standard monopolar electrocautery. Studies have shown that energy devices significantly reduce operating times without increasing complications or costs [36].

However, a systematic review by Hua et al. found no substantial differences in the rates of post-thyroidectomy hematoma when comparing alternate energy instruments to conventional hemostasis methods such as bipolar and monopolar cautery, "clamp-and-tie," or vascular ligations [37].

Hemostatic agents: During thyroid surgery, it is not uncommon to encounter minor, persistent bleeding from the superior pedicle or the area adjacent to the recurrent laryngeal nerve. However, using any of the aforementioned methods to manage this type of bleeding may significantly increase the risk of nerve injury. The use of adjunctive hemostatic agents in such cases has been investigated in numerous studies.

Surgicel is an oxidized cellulose mesh that adheres to tissue and aids in the formation of a hemostatic clot, particularly in bleeding areas. In 2013, Amit et al. found that the Surgicel group had significantly higher postoperative drain output (133 vs. 93 mL), delayed drain removal time (1.87 vs. 1.4 days), and a longer hospital stay (2.7 vs. 1.8 days) compared to the control group [38]. In another study by Testini et al., the use of FloSeal or a cellulose patch intraoperatively was compared to conventional surgery alone. The study included 155 subjects, 49 undergoing surgery alone, 52 receiving a cellulose patch, and 54 receiving FloSeal. Patients who underwent surgery with the cellulose patch or surgery alone had significantly longer operative times, time to drain removal, and hospital stays. However, there were no differences between the three groups in terms of postoperative hematoma or other complications of thyroid surgery [39]. In a different study, Docimo et al. reported that the group of patients given FloSeal in combination with Harmonic scalpel showed significantly lower drain output volumes in the first 24 hours compared to the group receiving conventional treatment (48.1 vs. 97.9 mL) [40].

Karanikolic et al. conducted a randomized study comparing the efficacy of three different hemostatic modalities in terms of blood loss, operative time, drainage volume, hospital stay, and postoperative complications. Patients were randomized into one of three groups: Group I used classic surgical procedures for hemostasis; Group II used a cellulose-based hemostat (Surgicel); and Group III used a fibrin-based hemostat (Beriplast). The study found that the use of the fibrin-based hemostat (Beriplast) resulted in a statistically significant reduction in surgical time, intraoperative blood loss, time to drain removal, and postoperative hospital stay compared to both traditional procedures and the cellulose-based hemostat (Surgicel). However, there were no significant differences in postoperative complications among the groups. The study suggested that fibrin-based hemostats should be used as a first-line hemostatic agent in thyroidectomy in combination with conventional surgical means of hemostasis [41].

In a descriptive retrospective study by Scaroni et al., the use of TachoSil (fibrinogen and thrombin-coated matrix) was associated with a trend toward less postoperative bleeding. The combination with other patches did not appear more effective [42]. In a small randomized controlled pilot trial, patients on antithrombotic medications still had a higher incidence of postoperative bleeding despite the use of TachoSil [43].

Strap muscle closure: How the strap muscles are closed can help reduce certain risks associated with postoperative hematoma. Traditionally, these muscles have been reapproximated from top to bottom using absorbable sutures. However, due to the association between airway obstruction and postoperative bleeding, which can obstruct lymphatic and venous outflow, many surgeons now prefer a single-point repair of the strap muscle diastasis. Placing a figure-of-eight absorbable suture at the midpoint of the strap muscles can potentially mitigate the risk of catastrophic airway obstruction. Another approach to achieving a similar goal is to use interrupted sutures, leaving the inferior part of the midline open to allow for possible drainage of a central neck hematoma. Some surgeons choose not to close the strap muscles in patients with thick necks [2].

Intraoperative Valsalva maneuver and Trendelenburg's positioning: Various techniques can assess intraoperative hemostasis. The most commonly performed techniques include Trendelenburg's positioning and the Valsalva maneuver, which aim to raise venous pressure and expose bleeding vessels.

Friedrich Trendelenburg originally described Trendelenburg's position as a technique to improve the surgical field of view during laparotomy. It was also considered a measure to enhance cardiac output in hypovolemic patients. Trendelenburg's positioning raises mean arterial pressure [44]. According to a study conducted by Rex et al., the optimal tilt angle for an appropriate increase in the size of the internal jugular vein during Trendelenburg's positioning was found to be 30 degrees [45]. However, this technique may be limited by the risk of increased intracranial pressure. Ozdemir et al. found that the tilt alone identified 47% of bleeding points [46]. Maintaining Trendelenburg's position for more than one minute is not recommended. This maneuver is overly sensitive in detecting bleeding vessels, as reported by Moumoulidis et al. [47].

The Valsalva maneuver is associated with increased intra-abdominal pressure, hemodynamic changes, and a rise in blood pressure [48]. The Valsalva maneuver is believed to assist in hemostasis during surgery by raising internal jugular vein pressure [49]. However, the Valsalva maneuver has limitations as it requires increased positive expiratory pressure, which carries the risk of pneumothorax. Therefore, it is recommended not to perform this maneuver for more than one minute [47]. It is well understood that venous pressure increases in the jugular veins when the Valsalva maneuver is combined with Trendelenburg's positioning [50]. A study by Ozdemir et al. revealed that the Valsalva maneuver effectively identified additional bleeding sites in Trendelenburg's position, increasing the detection of bleeding sites from 47% to 86.5% [46].

Deep extubation: When a patient emerges from anesthesia, deep extubation is a beneficial technique following endocrine neck surgery. Performing extubation under deep anesthesia reduces the occurrence of coughing and straining on the breathing tube, thereby minimizing cardiovascular stimulation. However, deep extubation may not be suitable for patients with specific conditions such as morbid obesity, airway pathology, gastroesophageal reflux, obstructive sleep apnea, and others who experience difficulties during intubation [2].

Pressure dressing: A randomized controlled trial conducted by Piromchai et al. examined the effect of pressure dressing on postoperative fluid collection. In this study, a total of 116 thyroidectomy patients were randomly allocated to either a non-pressure dressing group or a pressure dressing group. Researchers used ultrasound to assess the amount of fluid accumulation in the postoperative period. The findings of the study revealed that the group with pressure dressings had a lower level of drainage and fluid collection in the surgical bed. However, the difference was not statistically significant enough to recommend the routine use of pressure dressings. Nonetheless, some experts hypothesize that pressure dressings may delay the detection of hematomas due to the widely covered area of the neck [51].

Adrenaline spray: Adrenaline spray is commonly employed to minimize intra- and postoperative bleeding in various surgical fields [52-53]. However, the effectiveness of adrenaline spray in the context of thyroid surgery has not been well established. To address this gap, Ersoy et al. conducted a randomized controlled trial involving 80 patients to investigate the benefits of adrenaline spray in preventing postoperative bleeding after thyroid surgery. The study found that in the group of patients who received adrenaline, the mean amount of drainage was 36.65 ml, whereas in patients who did not receive adrenaline, the mean amount of drainage was 51.75 ml. This difference was statistically significant. However, limitations such as restricted sample size and the absence of postoperative hematoma and wound infection make the results inconclusive [54].

Drains: Drains were commonly used in thyroid and parathyroid operations, but their usage has declined due to multiple studies, including randomized trials, evaluating their effectiveness in preventing postoperative hematomas [55,56]. Most of these studies found no benefits in using drains to prevent hematomas, and surprisingly, some reports even indicated an increase in postoperative morbidity associated with their use [55]. In an analysis of 150 patients, Hurtado-Lopez et al. found that factors such as gland size, type of surgery, diagnosis, and intraoperative bleeding did not justify the use of external drains [57]. A systematic review published in 2017 comparing the use of drains versus no drains in thyroid operations concluded that drains did not reduce the risk of hematoma or seroma formation, nor did they reduce the risk of reoperation [56]. This finding aligns with previous meta-analyses [58,59].

Conversely, drains were associated with an increased risk of wound infection, postoperative pain, and prolonged hospital stays. Some studies even suggest that drains may contribute to increased fluid collection [57,60]. Furthermore, a prospective study by Al-Qahtani and Osman demonstrated that routine drainage did not significantly prevent post-thyroidectomy bleeding but did prolong hospital stays [61].

Table 2 summarizes the different strategies proposed for preventing bleeding after thyroid surgery.

**Table 2:** Different strategies proposed for the prevention of bleeding after thyroid surgery

Timing	Strategy
Preoperative considerations	Management of anticoagulation
Intraoperative considerations	Potentially beneficial:
	Anesthesia: minimize nausea - smooth emergence
	Surgical technique: conventional hemostasis techniques - alternate energy instruments
	Hemostatic agents: use of adjunctive hemostatic agents for minor bleeding or oozing near important structures
	Strap muscle closure: single-point repair - leaving the inferior part of the midline open
	Valsalva Maneuver and Trendelenburg's positioning: raising venous pressure to expose bleeding vessels
	Deep extubation: decreases coughing and straining
	No proven benefit:
	Pressure dressing
	Adrenaline spray
	Drains

Various protocols have been suggested to prevent and manage neck hematomas. Edafe et al. proposed a step-wise approach, known as the ITSRED Fred protocol, to reduce bleeding risk and aid in the early detection and management of bleeding following parathyroid and thyroid surgery (SCOOP protocol) [33].

## Conclusions

Compressive neck hematoma is a rare yet devastating complication of thyroid surgery. Thorough preoperative risk stratification, careful perioperative optimization, and prompt postoperative recognition and management are paramount for the safe and successful performance of thyroid surgery.
